The article "Prediction Model of Soil Heavy Metal Content Based on Particle Swarm Algorithm Optimized Neural Network" was published in 2022. Journal: Comput Intell Neurosci.

# Prediction Model of Soil Heavy Metal Content Based on Particle Swarm Algorithm Optimized Neural Network

**DOI:** 10.1155/2022/9693175

**Published:** 2022-09-02

**Authors:** Cuiqing Duan, Baoqiang Wang, Jinxiu Li

**Affiliations:** ^1^School of Environmental and Municipal Engineering, Lanzhou Jiaotong University, Lanzhou 730070, China; ^2^Gansu Academy of Social Sciences, Lanzhou 730070, China; ^3^Gansu Agricultural University, Lanzhou 730070, China

## Abstract

In 2014, the relevant research data from the Ministry of Environmental Protection and the Ministry of Land and Resources showed that the total exceedance rate of soil heavy metal pollution in China had reached 16.1%, and in the construction of ecological civilization in the 13th Five-Year Plan, China has made the prevention and control of soil heavy metal pollution as the focus of prevention and control. Therefore, in this paper, four neural optimization network models, that is, radial basis neural network (RBFNN), generalized regression neural network (GRNN), wavelet neural network (WNN), and fuzzy neural network (FNN), are simulated and created to measure and correlate the soil heavy metal content in a city in northwest China and a city in central China from the actual situation in China. The simulations were conducted. Finally, by analyzing the comparison of predicted and true values of these four models on the test data of two sets of experimental data, the distribution of predicted differences to true values, and the calculation results of three error indicators, we found that WNN has the best prediction performance when using RBFNN, GRNN, WNN, and FNN for soil heavy metal content prediction.

## 1. Introduction

The current situation of soil heavy metal pollution in China is still in a very serious state, especially with the rapid development of industrialization and urbanization, the emission of heavy metal pollution will continue to grow in the coming period of time, and this pollution will also be absorbed by human body with the material cycle of nature, which directly endangers human health. As early as 2014, the Ministry of Environmental Protection and the Ministry of Land and Resources showed that the total exceedance rate of soil heavy metal pollution in China had reached 16.1%, and in the 13th Five-Year Plan for the construction of ecological civilization, China has made the prevention and control of soil heavy metal pollution a priority [1].

The treatment of soil heavy metal pollution often needs to be tailored to local conditions, and it is necessary to fully understand the information on the content of various heavy metals in the contaminated area, and the main way to obtain this information is through field sampling and testing by researchers [2]. However, in the actual sampling process, due to the large area to be monitored, it is often difficult to collect every area, and because of the tedious process of soil heavy metal content testing and the large number of heavy metal categories to be tested, when the number of sampling points exceeds a certain number, the time and manpower required for testing will also be too high. Therefore, in order to obtain more detailed information about the soil heavy metal content, researchers usually use the soil heavy metal content data from some sampling points to predict the soil heavy metal content in other unknown areas, so as to obtain more abundant data information for decision making.

The article "Prediction Model of Soil Heavy Metal Content Based on Particle Swarm Algorithm Optimized Neural Network" was published in 2022. Journal: Comput Intell Neurosci.

The traditional data prediction methods can achieve good prediction results when dealing with data with a large number of features, but once the number of features decreases, the prediction performance also decreases. For example, in the source project of this thesis, the soil heavy metal content dataset obtained through the collection only contains five types of features: longitude, latitude, elevation, functional area, and eight heavy metals, and the number of features is relatively small. Therefore, it is difficult to obtain good prediction results when using traditional data prediction methods. With the continuous development of artificial intelligence in recent years, artificial neural networks have been increasingly used for data prediction in various industries, such as house price prediction, electricity load prediction, and short-time traffic flow prediction [3]. It has been proved to have better mapping ability and self-learning capability when dealing with data sets with complex nonlinear relationships, while the method can still achieve better prediction results when the relevant features in the training data are fewer or less relevant; for example, in the literature, researchers used only three types of feature data, namely, ambient temperature, daily average solar irradiation intensity, and daily average wind speed, as the BP neural network input to predict the output power of PV plants, and the average absolute percentage error of the predicted values is 28.4%, which is a relatively good result [4]. In addition, the application of artificial neural network in soil heavy metal content prediction is relatively small, and conducting related research can further verify the effectiveness of artificial neural network in data prediction, so this study chooses to use artificial neural network as the basic model for soil heavy metal content prediction research [5].

## 2. Research Background

At present, researchers' research on soil heavy metal content mainly involves several aspects such as pollution analysis of soil heavy metal content, spatial distribution study of soil heavy metal content, and prediction of soil heavy metal content, but when conducting pollution analysis of soil heavy metal content and spatial distribution study, they all involve prediction of soil heavy metal content in unknown areas, so soil heavy metal content prediction study is an, therefore, important part of soil heavy metal content research [6].

The article "Prediction Model of Soil Heavy Metal Content Based on Particle Swarm Algorithm Optimized Neural Network" was published in 2022. Journal: Comput Intell Neurosci.

In a foreign study on pollution analysis of soil heavy metal content, Susana et al. used geographically weighted principal component analysis to assess the diffuse sources of soil heavy metals and finally identified two major sources, which were geological causes related to mining and atmospheric causes related to vegetation burning [7]. Ha et al. used principal component analysis (PCA) to characterize the distribution of heavy metals in soil, then used kriging interpolation for the creation of regional distribution maps, and finally analyzed the distribution of soil heavy metal content and pollution in the target area using its better linear unbiased estimation; after visualizing the distribution of heavy metal pollution levels in urban soils, Jia et al. established artificial neural networks with reference to knowledge analysis of the causes of pollution as a way to determine the main causes of urban soil heavy metal pollution [8]. Ma et al. applied machine learning algorithm to soil heavy metal pollution analysis and established three prediction models, namely, support vector Machine (SVM), random forest (RF), and extreme learning machine (ELM), respectively, through correlation analysis of heavy metal content. In comparison with the experimental results, it was found that the concentration of soil heavy metal samples had a direct influence on the prediction effect of the model [9].

In the spatial distribution of soil heavy metal content and soil heavy metal content prediction research, Mr. Pandit and others used reflection spectroscopy to measure the reflectivity of different heavy metals, and then, by using partial least squares (PLSR) model to reflect the relationship between the soil heavy metal content and high spectral reflectance, the soil heavy metal content is predicted according to [10]. Aryafar et al. used support vector machine (SVM) to evaluate soil heavy metal pollution in the target river region and compared the prediction results of SUPPORT vector machine with the generalized regression neural network (GRNN). The results showed that the prediction accuracy of heavy metal content of SUPPORT vector machine was higher than that of the generalized regression neural network [11]. Naderi et al. established soil heavy metal distribution models based on stepped-multiple linear regression (MSLR) and genetic algorithm-optimized neural network (ANN-GA), respectively, and then compared soil heavy metal estimation results of the two models. It is proved that the latter method of using intelligent algorithm to optimize artificial neural network parameters has higher prediction accuracy [12].

The article "Prediction Model of Soil Heavy Metal Content Based on Particle Swarm Algorithm Optimized Neural Network" was published in 2022. Journal: Comput Intell Neurosci.

In the domestic research on pollution analysis of soil heavy metal content, Maimaititurson Aizezi et al. first used geostatistical method to analyze the spatial distribution of soil heavy metal content in the study area and then used two pollution evaluation indexes to evaluate the degree of soil heavy metal pollution in the region. It is determined that the main influencing sources of soil heavy metal content in this region are soil geochemical genesis and human activities [13]. Lin Xiaomei et al. chose least squares support vector machine (LSSVM) and partial least squares method (PLS) as comparative methods and combined them with induction technology, respectively, to conduct comparative experiments on soil heavy metal analysis. The results showed that the least squares support vector machine performed better in model accuracy and stability [14]. Wang Mudong et al. combined BP neural network and principal component analysis when analyzing the content of heavy metals in the soil of oil mining areas. The former was used to supplement the missing data in the experiment, and the latter was used for source analysis. Finally, they learned that the main sources of heavy metals in the soil were nature, agriculture, transportation, and coal burning [15]. In terms of the spatial distribution of soil heavy metal content, Jiang Zhenlan et al., based on geographical weighted regression (GWR) model, applied hyperspectral prediction of soil heavy metal content and compared the prediction results with OLS. The results showed that the geographical weight regression model could well reveal the spatial heterogeneity of the relationship between soil heavy metal content and related variables while having higher prediction accuracy [16]. Bayesian maximum entropy (BME) was applied to the spatial prediction of soil heavy metal content by Fei Xufeng et al. Compared with the ordinary Kriging interpolation method, the prediction error of this method is smaller, which can effectively help researchers determine the spatial distribution of soil heavy metal content [17]. In terms of the prediction of heavy metal content in soil, Gao Wenwu et al. first used variance analysis to determine the impact of different cultivated land types on heavy metal Mn in soil and then used collaborative Kriging interpolation to predict the content of Mn. Three error indicators, such as the average error, in the experimental results were all at low values. This indicates that the method has a high prediction accuracy for Mn content in soil [18]. Fan Junnan et al. used the applications of BP neural network model to predict soil heavy metal content, using the model of soil spatial location and the nonlinear mapping relationship between different heavy metals, to predict the heavy metal content of the value obtained in the use of simulation efficiency coefficient (NSE) to evaluate reliability prediction results after coming to the conclusion that the NSE value satisfies the requirement of simulation precision of the model, It has a good prediction effect [19]. Qin Xichun used three kinds of neural networks, respectively, to predict soil heavy metal content in his study. Through the comparison of experimental results, it was found that the prediction error of BP neural network was the largest among the three kinds of neural networks, while the errors of wavelet neural network (WNN) and radial basis neural network (RBFNN) were relatively close [20]. Therefore, based on relevant theories, this paper established four models needed in this paper to predict soil heavy metal content, evaluate the advantages and disadvantages of the models, and select the best model.

The article "Prediction Model of Soil Heavy Metal Content Based on Particle Swarm Algorithm Optimized Neural Network" was published in 2022. Journal: Comput Intell Neurosci.

## 3. Basic Theories and Research Methods

### 3.1. Basic Theory

#### 3.1.1. Theory of Soil Heavy Metal Content Measurement

There are many theories about soil heavy metal content measurement at home and abroad, and the measurement methods are abundant and involve a wide range. In metrology, mathematics, statistics, computer, and other disciplines are used to establish a wide range of models, which provides great support for the theoretical research of this paper. Therefore, in this paper, four neural optimization network models including radial basis neural network (RBFNN), generalized regression neural network (GRNN), wavelet neural network (WNN), and fuzzy neural network (FNN) were created to study soil heavy metal measurement methods. This paper focuses on the study and measurement of the following six heavy metals, as shown in Figure 1.

#### 3.1.2. Particle Swarm Algorithm Theory

Particle swarm optimization (PSO) algorithm is a new Evolutionary Algorithm (EA) developed in recent years. Dr. Eberhart and Dr. Kennedy were inspired by the regular clustering of birds in 1995 when they studied their predatory behavior. At first, a simplified model was established by using the idea of swarm intelligence, and then particle swarm algorithm was invented. On the basis of swarm intelligence, particle swarm optimization (PSO) makes use of the information exchange and sharing among individuals, so that the movement of the whole group can produce an orderly evolution process in the problem-solving space and then obtain the optimal solution. It has been widely used in the optimization of complex functions, neural network training, and other applications of evolutionary algorithms.

The article "Prediction Model of Soil Heavy Metal Content Based on Particle Swarm Algorithm Optimized Neural Network" was published in 2022. Journal: Comput Intell Neurosci.

The training process of particle swarm optimization: particle swarm optimization (PSO) randomly starts a set of solutions for each particle and then gradually updates and optimizes them through iterative algorithm. In each iteration, each particle updates its velocity and position by chasing two extremes. An extremum is the optimal solution previously found by the particle, and this extremum is called individual extremum pBest. The other extreme is the optimal solution currently found by the whole population. This extreme is called the global extreme gBest. In addition, gBest can not use the extreme value of the whole population, but only the individual extreme value nBest of the particles in the neighborhood within a certain range of the particle. Such particle swarm is the local version of the particle swarm, and the spatial topological structure of the particle determines the range of the neighborhood.

PSO algorithm is a global search algorithm, which randomly initializes many particles evenly distributed throughout the solution space. These particles carry out iterative search in the global space by combining their own and global information through certain strategies, and it will have a high probability to find a better solution:

1. *Global Particle Swarm*. If we update gBest each time looking for the best fit of all contemporary particles, then such a particle swarm is a global particle swarm. Global particle swarm is a bit greedy in nature, so its advantage is fast convergence speed, and its disadvantage is being easy to fall into the local optimal solution.
2. *Local Neighborhood Particle Swarm*. If we update gBest, we can choose a neighborhood K. For each particle, we update gBest according to the particle with the best fitness among the K particles around it. Because the similar particles have more similar properties, the local optimum can be replaced by the global optimum, so that the whole particle swarm can keep strong searching ability. Therefore, its advantages are having a stronger search range and being easy to jump out of the local optimal, and the disadvantage is also obvious, that is, slow convergence.
3. *Local Random Particle Swarm*. If K particles can be randomly selected when updating gBest, we will update gBest according to the particle with the best fitness among the K particles. We know that close particles have more similar properties, and if one particle deviates from the optimal solution, then several particles around it may deviate, so that their local optimal may not be very helpful for the whole population to find the optimal solution. Selecting K particles at random (the particles themselves should be kept) gives a certain probability of weeding out the bad ones. Therefore, it is a compromise between maintaining the searching ability and convergence speed of the whole population.

The article "Prediction Model of Soil Heavy Metal Content Based on Particle Swarm Algorithm Optimized Neural Network" was published in 2022. Journal: Comput Intell Neurosci.

#### 3.1.3. Particle Swarm Optimization Neural Network

With the optimization objective, the parameters of particle swarm optimization algorithm are determined. If the fitness function is known, the particle swarm optimization algorithm can be directly used to replace the BP algorithm to train the convolutional neural network.

The determination of fitness function of particle swarm optimization algorithm: in the process of deriving the parameters of convolutional neural network above, we see that the loss value of a network training loss will be calculated in the last loss layer. SOFTMAX_LOSS is generally used in convolutional neural network. This value is the error of network training. The closer it is to 0, the better the current training model is. This value is directly taken as the adaptive value of PSO, and the adaptive function of PSO can also be used to calculate the forward process of loss by convolutional neural network. After decoding the particle, the corresponding network structure weight can be obtained, and then the input sample is input into the network, and the forward process calculation is carried out with the network weight, and the training error loss value can be obtained.

We have analyzed the codec of convolutional neural network and determined the parameters of particle swarm optimization. The fitness function of particle swarm optimization algorithm is the convolution neural network to calculate the Loss worth process, and the training error loss is the adaptation value of PSO. Given these conditions, we can use particle swarm optimization to train the convolutional neural network.

For small samples, all training can be divided into a group; that is, batch-size is equal to the number of training samples, which is equivalent to full-sample training mode. However, when the sample size increases, the data exchange between layers is also related to batch-size. Generally, the training of convolutional neural networks is run in GPU mode, and all data will be stored in video memory. Too large batch-size will lead to insufficient video memory space for training. Therefore, in the case of large-scale training samples, mini-batch training mode can only be adopted. Since the convolutional neural network is grouped by batch_size for BP training, different training samples with the same network parameters will calculate different loss values, and if our PSO does so, then this loss value has no reference value. Therefore, PSO must go through all groupings to calculate the adaptation value and then find the average loss, which is the final adaptation value. This also means that the PSO algorithm can be very slow in large-scale samples. In addition, we know that BP is a gradient descent algorithm, and the gradient descent algorithm is easy to fall into local optimum; PSO algorithm is a relatively global algorithm, which increases the search range by multiparticle common search, at the cost of its relatively weak local search ability, and it also falls into local optimum solution. Especially in the case of high dimension and high samples, the local optimal solution that PSO falls into may not be as good as BP, and the higher the dimension is, and the more the samples are, the more difficult it is for PSO to jump out of this solution. The optimization performance of the particle swarm algorithm on sample sets of different sizes will be highlighted in the later experimental analysis.

The article "Prediction Model of Soil Heavy Metal Content Based on Particle Swarm Algorithm Optimized Neural Network" was published in 2022. Journal: Comput Intell Neurosci.

### 3.2. Research Methods

#### 3.2.1. Radial Basis Neural Network

Radial Basis Function Neural Network (RBFNN) is the most typical three-layer forward neural network structure. In addition to the information processing of traditional neural networks, its implicit layer uses radial basis functions for nonlinear mapping of input data, which is then passed to the next layer after linear computation. The structure of the radial basis neural network is shown in Figure 2.

In the unsupervised learning part, the data are clustered by using a clustering algorithm such as K-means to obtain the centroid of the radial basis function in the hidden layer, and then the width vector of the radial basis function is calculated by using the centroid information, and the width vector is calculated by the following formula:

(1) $$\begin{array}{c} \sigma_{j}=\frac{c_{xy}}{\sqrt{2h}}\text{,} \end{array}$$

where *c*_*Xy*_ is the maximum distance before the centroid and *h* is the number of nodes.

After that, the input data are related to the scattering through the implicit layer and the output layer, respectively, and the output *x*_*i*_ of the first node *j* of the input sample in the implicit layer is calculated by the following equation:

(2) $$\begin{array}{c} \phi \left(x_{i},j\right)=\exp\left(-\frac{1}{2\sigma_{j}^{2}}x_{i}-c_{i}\right)\text{,} \end{array}$$

where *c*_*j*_ and *σ*_*j*_ are the centroid and width *m* vector of the first node in the hidden layer, respectively.

The article "Prediction Model of Soil Heavy Metal Content Based on Particle Swarm Algorithm Optimized Neural Network" was published in 2022. Journal: Comput Intell Neurosci.

The output of *x*_*i*_ the first node of *j* the input sample in the output layer is calculated by the following equation:

(3) $$\begin{array}{c} y_{m}=\varphi \left(\phi \left(x_{i},j\right)*w_{m}\right)\text{,} \end{array}$$

where *w*_*m*_ is the node weight and *φ* is the activation function.

In the supervised learning part, it is mainly the process of continuously correcting the parameters in each layer, and this process is mainly calculated by the error function to calculate the gradient value of each parameter, and then the parameters are continuously corrected using traditional gradient descent methods such as stochastic gradient descent (SGD); taking the weights used for linear calculation in the output layer as an example, the update formula is as follows:

(4) $$\begin{array}{c} w_{t}=w_{t-1}-u*\frac{\sigma E}{\sigma w_{t-1}}\text{,} \end{array}$$

where *E* is the error function and *u* is the learning rate

In addition to the above methods, the centroids and width vectors of the hidden layer can be directly generated randomly, after which they are updated according to the gradient correction formula of the supervised learning process.

#### 3.2.2. Generalized Regression Neural Network

Generalized Regression Neural Network (GRNN) is a four-layer forward propagation neural network with fewer parameters and better nonlinear mapping capability in its network structure [26][27], where the data are input to the network, and the output results are obtained after passing through the input layer, pattern layer, summation layer, and output layer in turn. This network does not have a training process but mainly optimizes the smoothing factor of the pattern layer to obtain good output results as shown in Figure 3.

The computational process is not shown in detail here, and the specific computational process can be obtained by the radial basis neural network inversion, which will not be done in this case. Although GRNN does not require network training, the smoothing factor of the pattern layer has a large impact on the performance of the network, and too large or too small smoothing factor will lead to underfitting and overfitting of the network, respectively, and it is usually difficult to set the smoothing factor to a better value in the experiment, so if you want to get better network performance, you generally choose an efficient intelligent optimization algorithm to find the optimal smoothing factor.

#### 3.2.3. Wavelet Neural Network

Wavelet Neural Network (WNN) has a three-layer structure, which is characterized by the use of wavelet basis function as the activation function of the neurons in the hidden layer, which makes the network more capable of self-learning when processing data sets with large amounts of data, so it can fit complex relational data faster. Its structure is shown in Figure 4.

The article "Prediction Model of Soil Heavy Metal Content Based on Particle Swarm Algorithm Optimized Neural Network" was published in 2022. Journal: Comput Intell Neurosci.

The computational process is not shown in detail here, and the specific computational process can be obtained by the radial basis neural network inversion, which will not be done in this example. There are four main parameters in WNN, and the size of these four parameter values will directly affect the performance of the network, so the training process of WNN as RBFNN mainly uses the traditional gradient descent method such as stochastic gradient descent (SGD) to continuously correct these four parameters.

#### 3.2.4. Fuzzy Neural Network

Fuzzy Neural Network (FNN) incorporates fuzzy theory into the information transfer process of the network, which can have a larger processing range and faster information processing speed when processing information, so the self-learning ability and mapping of the network are relatively high. The structure diagram of fuzzy neural network is commonly used and can be found in general textbooks, so it is not repeated in this paper.

The data is trained by this neural network through a total of five layers: the first is the input layer, and the number of nodes in this layer is related to the feature dimension of the data; that is, when the feature dimension of the data is *n*, the number of nodes in the input layer is *n*. Then, the data is passed from the input layer to the affiliation function calculation layer, where the affiliation function is used to calculate the affiliation of each node, each node represents an affiliation function, and the number of nodes in this layer is the number of possible fuzzy conditions of the input variables. When the dimensionality of the output variables increases, the weights will be adjusted accordingly. In addition, FNN, like the previous RBFNN and WNN, generally uses traditional gradient descent methods such as stochastic gradient descent (SGD) to optimize the centroids of the affiliation function, the width vector, and the connection weights of the output layer.

## 4. Research Results and Discussion

In order to compare the prediction performance of the above four artificial neural networks for soil heavy metal content prediction, the authors will build models for each of the above four artificial neural networks and then choose the same soil heavy metal dataset for prediction experiments under the same experimental environment.

### 4.1. Selection and Preprocessing of Soil Heavy Metal Data

The first dataset is the surface soil heavy metal content dataset of an urban area in a provincial capital in Northwest China, which was sampled by the School of Resources and Environment of a university and is a publicly available dataset. This dataset contains the contents of a total of six heavy metals, namely, cobalt (Co), chromium (Cr), cesium (Cs), magnesium (Mg), lead (Pb), and titanium (Ti), and the total number of samples is 96 sets of these soil heavy metal content specifics.

The article "Prediction Model of Soil Heavy Metal Content Based on Particle Swarm Algorithm Optimized Neural Network" was published in 2022. Journal: Comput Intell Neurosci.

Among the specific cases, the minimum value of elemental cobalt (Co) was 16.7 mg per kg of soil; the maximum value was 108.4 mg per kg of soil; the mean value was 37.23 mg per kg of soil; and the standard deviation was 17.43 mg per kg of soil. The minimum value of elemental chromium (Cr) was 66.2 mg per kg of soil; the maximum value was 143.8 mg per kg of soil; the mean value was 109.07 mg per kg of soil; and the standard deviation was 12.79 mg per kg of soil. The minimum value of elemental cesium (Cs) was 0 mg per kg of soil; the maximum value was 42 mg per kg of soil; the mean value was 17.35 mg per kg of soil; and the standard deviation was 9.69 mg per kg of soil. The minimum value of magnesium (Mg) was 0.98 mg per kg of soil; the maximum value was 3.25 mg per kg of soil; the mean value was 2.13 mg per kg of soil; and the standard deviation was 0.4 mg per kg of soil. The minimum value of elemental lead (Pb) was 12.8 mg per kg of soil; the maximum value was 49.1 mg per kg of soil; the mean value was 24.99 mg per kg of soil; and the standard deviation was 5.41 mg per kg of soil. The minimum value of elemental titanium (Ti) was 1189 mg per kg of soil; the maximum value was 2441 mg per kg of soil; the mean value was 2040.23 mg per kg of soil; and the standard deviation was 341.14 mg per kg of soil.

Since this dataset contains a small amount of data, a total of 96 groups of data, no processing such as feature selection was performed on the dataset, and the content of heavy metal Co was selected as the feature to be predicted, and the other five heavy metals were used as the input feature data for the model. After that, 20 sets of data were randomly selected from this data set as the test data, and the rest of the data were used as the training data.

The second data set is the soil heavy metal data set of six new urban areas in a city in central China, which was collected and tested by the Institute of Environmental Safety of the Academy of Agricultural Sciences of a city in central China, one of the contractors of the source project of this study. We use Copper (Cu), Nickel (Ni), Lead (Pb), Zinc (Zn), and Mercury (Hg), giving the relevant situations of these eight heavy metals.

The article "Prediction Model of Soil Heavy Metal Content Based on Particle Swarm Algorithm Optimized Neural Network" was published in 2022. Journal: Comput Intell Neurosci.

Among the specific cases, the minimum value of elemental chromium (Cr) is 11.13 mg per kg of soil; the maximum value is 171.21 mg per kg of soil; the mean value is 57.49 mg per kg of soil; and the standard deviation is 24.64 mg per kg of soil. The minimum value of elemental arsenic (As) was 0.24 mg per kg of soil; the maximum value was 82.07 mg per kg of soil; the mean value was 10.15 mg per kg of soil; and the standard deviation was 6.00 mg per kg of soil. The minimum value of elemental cadmium (Cd) was 0.01 mg per kg of soil; the maximum value was 4.94 mg per kg of soil; the mean value was 0.21 mg per kg of soil; and the standard deviation was 0.39 mg per kg of soil. The minimum value of elemental copper (Cu) was 2.16 mg per kg of soil; the maximum value was 159.36 mg per kg of soil; the mean value was 26.21 mg per kg of soil; and the standard deviation was 14.06 mg per kg of soil. The minimum value of elemental nickel (Ni) was 3.32 mg per kg of soil; the maximum value was 77.67 mg per kg of soil; the mean value was 28.22 mg per kg of soil; and the standard deviation was 12.04 mg per kg of soil. The minimum value of elemental lead (Pb) was 1.96 mg per kg of soil; the maximum value was 83.30 mg per kg of soil; the mean value was 19.46 mg per kg of soil; and the standard deviation was 8.60 mg per kg of soil. The minimum value of elemental zinc (Zn) was 15.16 mg per kg of soil; the maximum value was 293.73 mg per kg of soil; the mean value was 71.17 mg per kg of soil; and the standard deviation was 29.29 mg per kg of soil. The minimum value of elemental Mercury (Hg) was 0.01 mg per kg of soil; the maximum value was 2.37 mg per kg of soil; the mean value was 0.14 mg per kg of soil; and the standard deviation was 0.17 mg per kg of soil.

This data set contains a total of 1161 sets of data, and 500 sets of sample data were randomly selected as experimental data. In data prediction experiments, when the correlation between the input features of the model and the features to be predicted is higher, the prediction effect of the model is better, and the correlation between heavy metals and heavy metals is often greater than the correlation between location information such as latitude and longitude and heavy metals. The Pearson coefficients between different heavy metals and heavy metal Cr were calculated, and according to the calculation results, the top five heavy metals with larger Pearson coefficients were As, Cd, Ni, Pb, and Zn selected as the input features of the model. After that, 50 sets of data were randomly selected from 500 sets of sample data as test data, and the remaining data were used as training data, and the prediction results of several models on 50 sets of test data were compared after training of the models. The Pearson coefficients of arsenic (As) were 0.5939; those of cadmium (Cd) were 0.3235; those of copper (Cu) were 0.1475; those of nickel (Ni) were 0.6652; those of lead (Pb) were 0.6356; the Pearson coefficient of zinc (Zn) is 0.4226, and the Pearson coefficient of Mercury (Hg) is 0.0411.

The article "Prediction Model of Soil Heavy Metal Content Based on Particle Swarm Algorithm Optimized Neural Network" was published in 2022. Journal: Comput Intell Neurosci.

### 4.2. Experimental Environment and Parameter Settings

In terms of parameter settings, the number of nodes per layer of the four network models needs to be determined first. Since the feature dimension of the input data is 5, and the feature dimension of the output data is 1 for both experimental data sets, the number of nodes and the feature dimension of the input and output layers of these four neural network models are the same, 5 and 1, respectively. The loss values of RBFNN and WNN vary irregularly with the change of the number of nodes in the hidden layer on either dataset, but the loss values of RBFNN and WNN are minimized when the nodes in the hidden layer are 7 and 8, respectively, so the number of nodes in the hidden layer is set to 7 and 8 for both datasets.

The RBFNN loss value and WNN loss value are both lower in a city in Northwest China again on each implied layer node tree, with a total of 11 nodes ranging from 2 to 12, and both loss values are above 2. The results show that the RBFNN loss value and WNN loss value are both lower in this city in Northwest China as shown in Figure 5.

The RBFNN loss value and WNN loss value are both higher for a city in central China than on each implied layer node tree, much higher than the northwest city selected in this paper with a total of 11 nodes from 2 to 12, and both loss values are about 6 or more, and the results show that the RBFNN loss value and WNN loss value are higher for the city in central China, and the contrast with the northwest city is obvious, as shown in Figure 6.

In GRNN, the number of nodes in the mode layer is the number of training dataset samples, then the number of nodes in the mode layer is set to 76 for the experiments on the Ningxia dataset, and the number of nodes in the mode layer is set to 450 for the experiments on the Wuhan dataset, so their corresponding numbers of nodes in the summation layer are 77 and 451, respectively. Since there is only one index to be predicted, we set the number of fuzzy conditions in FNN to 2. The number of fuzzy gradations for each sample feature in its subordination function calculation layer is 16; that is, the number of nodes in the rule generation layer and normalization layer is 16. GRNN has no training process, so a more appropriate smoothing factor value is selected for it according to the cross-validation method, while the other three neural networks are trained with the parameters of stochastic gradient descent method, and the number of training times of the network is set to 500, and the learning rate is set to the common 0.001.

The article "Prediction Model of Soil Heavy Metal Content Based on Particle Swarm Algorithm Optimized Neural Network" was published in 2022. Journal: Comput Intell Neurosci.

### 4.3. Experimental Results

After the training of the four neural network models was completed, their predicted and true values were first compared on the two data sets of the test set, and the graphs in this section show that there are points where the predicted and true values are the same, or the difference is larger for either neural network model, where the curve representing the predicted value of GRNN has a relatively low agreement with the curve representing the true value, as well as the curves representing the RBFNN, WNN, and FNN. The agreement between the curves representing the predicted values and the curves representing the true values is relatively high. Comparing the curves representing the predicted values of RBFNN, WNN, and FNN, we can see that the trends of these three curves are relatively close to each other. The main difference between a city in Northwest China and a city in Central China is that the curves of RBFNN and GRNN predictions are in relatively low agreement with each other than the curves representing the true values, while the curves representing WNN and FNN predictions are in relatively high agreement with the curves representing the true values. Therefore, it is difficult to see the difference between the prediction performance of these four neural networks from these two comparison graphs alone. In order to understand more clearly the difference between the predicted and true values of these four neural network models, the prediction difference value of each sample point in the test data set on the two experimental data sets will be calculated separately, and then the ratio situation between this difference value and the true value will be found, and finally the distribution of the 50 test data of the four neural network models in different ratio intervals will be counted. In order to have a clearer understanding of the difference between the predicted and true values of the four neural network models, the predicted difference values of each sample point in the test data sets of the two experimental data sets are calculated, and then, the ratio between the difference value and the true value is calculated, and finally the distribution of the 50 test data of the four neural network models in different ratio intervals is calculated, as shown in Figures 7 and 8.

The distribution of the ratio of the difference to the true value of the prediction data of different neural network models on the test data set of this city in the northwest shows a trend of low in the middle and high in the sides, in which it can be seen more obviously that the prediction model of this city in the northwest has a higher percentage of the true value and a higher accuracy rate as shown in Figure 7.

The article "Prediction Model of Soil Heavy Metal Content Based on Particle Swarm Algorithm Optimized Neural Network" was published in 2022. Journal: Comput Intell Neurosci.

The distribution of the ratio of the difference to the true value of the prediction data of different neural network models on the test dataset of this city in central China shows a trend of high left and low right, which shows that the prediction model in central China has a lower proportion of true values and a lower accuracy rate as shown in Figure 8.

In Figure 7, the distribution of points of FNN and GRNN is mostly concentrated in the range of less than 10% and more than 40%, and the number of their points greater than 40% is greater than the other two models, while the number of points of RBFNN and WNN in the range of less than 10% is slightly less than the other two models, but overall, the number of points of RBFNN and WNN in the range of difference ratio less than 30% is greater than the other two models. The number of points is more than the other two models. In Figure 8, the distribution of points of RBFNN is significantly smaller than that of the other three models in the interval of less than 10% and larger than that of the other three models in the period of 10% to 20%. The other three models are closer overall, but with 20% as the limit, the number of points of WNN in the interval less than 20% is larger than that of GRNN and FNN, and the number of points in the interval greater than 20% is smaller than them, while the number of points of GRNN and FNN is closer in these two intervals.

In addition to the comparison of the above two experimental results, the mean absolute error (Mean Absolute Error, or MAE), root mean square error (Root Mean Square Error, or RMSE), and symmetric mean absolute percentage error (Symmetric Mean Absolute Percentage Error), the smaller the calculated results of these three error indicators, the better the prediction performance of the model.

From the calculated results, we can understand that the main difference is that the values of the three error metrics of GRNN on the Ningxia test dataset are larger than those of the other three models, while the error metrics of RBFNN on the Wuhan test dataset have the largest values except for the RMSE values. However, the values of the three error indicators of WNN are smaller than those of the other three models in either test dataset, where the calculated results of WNN in the Ningxia test dataset are lower by about 2.8 mg/kg for MAE, 4.5 mg/kg for RMSE, and 7% for SMAPE compared with the maximum values of the three indicators. Compared with the maximum value of these three indexes, the MAE value is reduced by about 1.3 mg/kg, RMSE value is reduced by about 1.7 mg/kg, and SMAPE is reduced by about 2%. Combining the above three experimental results and analysis, it can be concluded that WNN has the best prediction performance when using the four neural networks RBFNN, GRNN, WNN, and FNN for soil heavy metal content prediction.

The article "Prediction Model of Soil Heavy Metal Content Based on Particle Swarm Algorithm Optimized Neural Network" was published in 2022. Journal: Comput Intell Neurosci.

## 5. Conclusion

In this paper, we first introduced the basic principles of four common neural networks and then modeled these four neural networks and compared their prediction performance in soil heavy metal content prediction. In this paper, four neural optimization network models, Radial Basis Neural Network (RBFNN), Generalized Regression Neural Network (GRNN), Wavelet Neural Network (WNN), and Fuzzy Neural Network (FNN), are simulated to measure and calculate the soil heavy metal content in a city in Northwest China and a city in Central China, using particle swarm algorithm. Finally, by analyzing the predicted and true values of these four models on the test data of two sets of experimental data, the distribution of the predicted difference to the true value, and the calculation results of three error indicators, we can find the prediction of soil heavy metal content using RBFNN, GRNN, WNN, and FNN neural networks.

This process includes the selection and preprocessing of experimental data, the setting of experimental environment and model parameters, and the training and testing of the four models. Finally, by analyzing the comparison plots between the predicted and true values of these four models on the test data of the two sets of experimental data, the distribution of the predicted difference in proportion to the true value, and the calculation results of the three error indicators, it can be found that the prediction performance of the wavelet neural network is better than that of the other three neural networks when performing soil heavy metal content prediction.

## Figures and Tables

**Figure 1:** Main types of heavy metals in soil.

**Figure 2:** Structure of radial basis neural network.

**Figure 3:** Structure of generalized regression neural network.

**Figure 4:** Structure of wavelet neural network.

**Figure 5:** Loss values of RBFNN and WNN on the dataset of this city in Northwest China.

**Figure 6:** Loss values of RBFNN and WNN on the Han dataset in central China cities.

**Figure 7:** Distribution of the ratio of the difference to the true value of the prediction data of different neural network models on the test dataset of the city in Northwest China.

The article "Prediction Model of Soil Heavy Metal Content Based on Particle Swarm Algorithm Optimized Neural Network" was published in 2022. Journal: Comput Intell Neurosci.

**Figure 8:** Distribution of the proportion of the difference to the true value of the predicted data of different neural network models on the test dataset of this city in central China.

## Data Availability

The dataset is available upon request.
